The article "Characterization of Vascular plant One-Zinc finger (VOZ) in soybean (Glycine max and Glycine soja) and their expression analyses under drought condition" was retracted in 2023. Reasons: a conflict of interest; concerns about the peer review; concerns about the authorship.

# Characterization of Vascular plant One-Zinc finger (VOZ) in soybean (*Glycine max* and *Glycine soja*) and their expression analyses under drought condition

**DOI:** 10.1371/journal.pone.0253836

**Published:** 2021-07-02

**Authors:** Shoaib Ur Rehman, Ghulam Qanmber, Muhammad Hammad Nadeem Tahir, Ahsan Irshad, Sajid Fiaz, Furqan Ahmad, Zulfiqar Ali, Muhammad Sajjad, Muhammad Shees, Muhammad Usman, Zhide Geng

**Affiliations:** 1 Institute of Plant Breeding and Biotechnology, Muhammad Nawaz Shareef University of Agriculture Multan, Multan, Pakistan; 2 State Key Laboratory of Cotton Biology, Cotton Research Institute of Chinese Academy of Agricultural Sciences, Anyang, Henan, China; 3 Institute of Crop Sciences, Chinese Academy of Agricultural Sciences, National Engineering Laboratory of Crop Molecular Breeding, National Center of Space Mutagenesis for Crop Improvement, Beijing, China; 4 Department of Plant Breeding and Genetics, The University of Haripur, Haripur, Pakistan; 5 Institute of Crop Science, College of Agriculture and Biotechnology, Zhejiang University, Hangzhou, China; 6 Department of Biosciences, COMSATS University Islamabad (CUI), Islamabad, Pakistan; 7 Institute of Food Crops, Yunnan Academy of Agricultural Sciences, Kunming, China; University of Education Lahore, PAKISTAN

## Abstract

Vascular plant one-zinc-finger (*VOZ*) transcription factors regulate plant growth and development under drought conditions. Six *VOZ* transcription factors encoding genes exist in soybean genome (both in *Glycine max* and *Glycine soja*). Herein, *GmVOZs* and *GsVOZs* were identified through *in silico* analysis and characterized with different bioinformatics tools and expression analysis. Phylogenetic analysis classified *VOZ* genes in four groups. Sequence logos analysis among *G*. *max* and *G*. *soja* amino acid residues revealed higher conservation. Presence of stress related *cis*-elements in the upstream regions of *GmVOZs* and *GsVOZs* highlights their role in tolerance against abiotic stresses. The collinearity analysis identified 14 paralogous/orthologous gene pairs within and between *G*. *max* and *G*. *soja*. The *Ka/Ks* values showed that soybean *VOZ* genes underwent selection pressure with limited functional deviation arising from whole genome and segmental duplication. The *GmVOZs* and *GsVOZs* were found to express in roots and leaves at seedling stage. The qRT-PCR revealed that *GmVOZs* and *GsVOZs* transcripts can be regulated by abiotic stresses such as polyethylene glycol (PEG). The findings of this study will provide a reference to decipher physiological and molecular functions of *VOZ* genes in soybean.

## Introduction

Wild soybean (*Glycine soja*) is an ancestor of cultivated soybean (*Glycine max* L.). Soybean is an important source of edible oil, protein, food, and feed [1]. Owing to intensive domestication and selection for higher yield, *G*. *max* has lost considerable genetic diversity through continuous genetic bottleneck. *G*. *soja* can be a promising source of new genes for *G*. max breeding required in response against climatic changes. The genomes of *G*. *max* and *G*. *soja* have been sequenced which enable whole genome analyses of gene families in both the species of soybean [2, 3].

The article "Characterization of Vascular plant One-Zinc finger (VOZ) in soybean (Glycine max and Glycine soja) and their expression analyses under drought condition" was retracted in 2023. Reasons: a conflict of interest; concerns about the peer review; concerns about the authorship.

Isolation and genome-wide characterization of plant transcription factors (TFs) have critical importance [4–6]. TFs play their role in stress tolerance by regulating stress responsive genes. Hence, expression of genes plays important roles in plant responses to different stimuli. Vascular plant one-zinc-finger (*VOZ*) TF family is present in many plant species. The *VOZ* family contains ~635 members and there homologous in 166 plant species [7]. The *VOZs* play protective role against ever changing environmental stresses and regulate plant growth and development. The VOZ proteins are plant specific TF family with two members, *VOZ1* and *VOZ2*, exclusively present in vascular plants [11]. Mitsuda et al. [8], identified the first VOZ protein which binds to the GCGTNx7ACGC palindromic sequence in the regulatory region of the *Arabidopsis thaliana* V-PPase gene (*AVP1*) using yeast one-hybrid screening [9–11]. This *VOZ* plays important role in regulating flowering in crop plants. The *VOZ1*/*2* phytochrome B-interact with TF and regulate the vegetative growth to reproductive stage by up-regulating flowering locus *T* and down-regulating flowering locus *C* expression in *A*. *thaliana* [12]. The *VOZ1*/*2* promote flowering mainly by modulating and interacting with *CONSTANS* (*CO*), though this is independent of *FLC* in *A*. *thaliana* [11]. Besides flowering, transcriptional regulators inhibits plant tolerance to abiotic stress factors such as drought, high and low temperature. For example, over-expression of *VOZ2*, damaged the tolerance of plants against drought and low temperature stresses in *A*. *thaliana* but improved resistance against fungal pathogen [13]. In *A*. *thaliana voz1/voz2* (dual mutants) showed enhanced tolerance to low temperature and water stresses. *VOZ1* and *VOZ2* suppressed the expression of *DREB2C* or *DREB2A* [14, 15]. During salt stress, *VOZ* also response likewise in low temperature and water stress conditions. According to some reportsthe genes, responsible for salt stress tolerance, are being controlled directly or indirectly by *VOZ1/2* [16, 17].

The article "Characterization of Vascular plant One-Zinc finger (VOZ) in soybean (Glycine max and Glycine soja) and their expression analyses under drought condition" was retracted in 2023. Reasons: a conflict of interest; concerns about the peer review; concerns about the authorship.

At first, *VOZ* gene family was characterized in *A*. *thaliana* based on its expression and function. Afterwards this gene family was reported in various crop plants [10, 16, 17]. Research on the characterization of *VOZ* in other crop species is still nascent. In this study, 12 members of *VOZ* family were characterized in *G*. *max and G*. *soja*. Phylogenetic analysis, sequence logos, sub-cellular localization, gene duplication chromosomal distribution, *Ka/Ks* ratio, promoter *cis*-element, and exon/intron structure were predicted. Moreover, sub-cellular localization and transcript abundance of *GmVOZs* and *GsVOZs* were also measured under drought stress conditions. The results of this study will provide a reference for future research on regulatory roles of VOZ transcription factors in soybean.

## Materials and methods

### Sequence identification

*Arabidopsis* VOZs protein sequences has been used as query sequences to identify *VOZ* transcription factors and proteins in different plant species such as *G*. *max*, *G*. *soja*, *M*. *truncatula*, *G*. *raimondaii*, *S*. *melongena*, *P*. *trichocarpa*, *P*. *patens*, *A*. *comosus*, *O*. *sativa*, *Z*. *mays* and *B*. *rapa*. To confirm the retrieved VOZ protein sequences, Interproscan 63.0 (IPR039277) (http://www.ebi.ac.uk/InterProScan/) and SMART (http://smart.embl-heidelberg.de/) tools were used. The identified VOZ members were confirmed by using Batch Web CD search tool CDD (Conserved Domains Database) search (https://www.ncbi.nlm.nih.gov/Structure/bwrpsb/bwrpsb.cgi). Biophysical properties such as protein length, isoelectric point, molecular weight were computed using ExPASy ProtParam tool (http://us.expasy.org/tools/protparam.html).

### Sequence alignment and phylogeny

To create sequence logos for conserved amino acid residues (AARs) multiple sequence alignment of *G*. *max* and *G*. *soja* was performed independently using CLUSTAL X 2.0 and sequence logos were created from WEBLOG [18]. For phylogenetic analysis, protein sequences of VOZs from different plant species were aligned and phylogenetic tree was made in MEGA V 6 (https://www.megasoftware.net) by using maximum likelihood (ML) method [19]. Bootstrap method with thousand replicates was used to determine the reliabilities of the groups.

### Sub-cellular localization

Sub-cellular localization of GsVOZs and GsVOZs were predicted using the online tool CELLOv.2.5 (http://cello.life.nctu.edu.tw/). The sub-cellular localization was also observed in *Nicotiana benthamiana* leaf cells having vectors with the coding regions of GmVOZ1 and GsVOZ1 and GFP as a control, were transferred into *N*. *benthamiana* leaves through *Agrobacterium tumefaciens* (GV3101) mediated transformation and spotted 4 days after incubation at 23°C in a photoperiod of 6 h dark and 16 h light. Oligonucleotide sequences and enzymes used in present study are provided in S1 Table.

The article "Characterization of Vascular plant One-Zinc finger (VOZ) in soybean (Glycine max and Glycine soja) and their expression analyses under drought condition" was retracted in 2023. Reasons: a conflict of interest; concerns about the peer review; concerns about the authorship.

### Exon/intron and *cis*-element analysis

*GmVOZs* and *GsVOZs* were initially aligned by CLUSTAL X 2.0 followed by MEGA V6 to create ML tree. The resultant bed-file was subjected to Gene structure display server 2.0 (GSDS), which was used to identify the exons and introns [20]. For *cis*-element analysis of *GmVOZs* and *GsVOZs* promoter regions ⁓2 kb upstream of ATG were considered as promoter region and subjected to PlantCARE Database [21] and predicted *cis*-element were categorized on the basis to their functional significance.

### Collinearity and *Ka/Ks* ratio analysis

For collinearity analysis, paralogous/orthologous data were obtained as descried by Yang et al. [22] and then figure was produced using CIRCOS package [23]. Non-synonymous (*Ka*) and synonymous (*Ks*) deviation level ratios were computed by aligning duplicated gene pair protein sequences in CLUSTAL X 2.0, after which they were translated into cDNA sequences using PAL2NAL program [24]. At the end, *Ka* and *Ks* values were computed with the help of CODMEL program using the PAML package [25].

### Gene expression profiling of *GmVOZs* and *GsVOZs*

*G*. *max* cv. William-82 and *G*. *soja* cv. W05 were used as plant material to determine the tissue specific expression pattern under normal as well as under drought stress conditions. To analyze the expression of *GmVOZs* and *GsVOZs* genes in different tissue and development stages, soybean plants were grown at research farm of MNS University of Agriculture, Multan, and all samples were collected under field conditions with standard agronomic practices. To explore the expression under drought conditions, William-82 and W05 were grown in a 3:1 (w/w) mixture of soil and sand (day/night temperature 22/20°C), germinated and irrigated with Hoagland solution once in every two days. After 28 days, the seedlings were germinated with 20% Poly Ethylene Glycol 6000 (PEG). Root samples from control and treated seedlings were taken at 0h, 1h, 3h and 6h after treatment. RNA was extracted using RNAprep Pure Plant Kit (TIANGEN, China). PrimeScript®RT reagent kit (Takara, China) was used to synthesize cDNA. For qRT-PCR, Premix Ex TaqTM II (Takara) was used and PCR amplification was performed on CFX connect Real-Time PCR detection system (Hercules, California 94547, U.S.A). The housekeeping genes, *Actin* and *GAPDH*, were used as internal control in *G*. *max* and *G*. *soja*, respectively. Each experiment was conducted in triplicates. Oligonucleotide sequences used in current work are listed in S1 Table.

The article "Characterization of Vascular plant One-Zinc finger (VOZ) in soybean (Glycine max and Glycine soja) and their expression analyses under drought condition" was retracted in 2023. Reasons: a conflict of interest; concerns about the peer review; concerns about the authorship.

## Results

### Identification of VOZ gene family members

*In silico* approach was used to identify the 47 *VOZ* gene members in 12 different species including 2 each from *Arabidopsis thaliana*, *Medicago truncatula*, *Brachypodium distachyon*, *Ananas comosus*, and *Solanum melongena*, 3 each from *Psychomitrella patens*, and *Gossypium raimondii*, 4 from *Populus trichocarpa*, 6 each from *Zea mays*, *Glycine max*, *Glycine soja* and 9 from *Brassica rapa*. We noticed that all the selected species have a minimum of two *VOZ* genes with *Z*. *mays*, *G*. *max*, *G*. *soja* and *B*. *rapa* have a greater number of members and *M*. *truncatula*, *P*. *paten* have only two and three members of *VOZ* genes, respectively, showing that this gene family was subjected to expansion in higher plants. The biophysical properties of *GmVOZ* and *GsVOZ* genes including locus ID, gene length, coding sequences (CDs), protein length, molecular weight (MW), isoelectric point (pI), chromosome position and sub-cellular localization of all *GmVOZs* and *GsVOZs* were determined (S2 Table). Fewer variations were observed in *GmVOZs* and *GsVOZs* in terms of coding sequences, proteins length and molecular weights. However, the predicted sub-cellular localization results indicated that all *GmVOZs* and *GsVOZs* are localized in nucleus (S2 Table).

### Sequence logos

Sequence logo was generated to check the extent of conserveness of VOZ proteins family in *G*. *max* and *G*. *soja* (Fig 1). We observed that sequence logos among two species were highly conserved across the N and C termini such as I (1), L (3), C (7)], P (8), F (9), L (10), W (26), H (32), F (55), and so forth (Fig 1). Beside this, no compositional bias of any pattern of conserved AARs was observed in sequence logos of *G*. *soja* and *G*. *max*. Sequence logos provides a defined depiction of sequence similarity as compared to consensus sequences, significant features of alignment, pattern in sequence conservation, and assist to discover and analyze those proteins [18]. Hence, VOZ sequence logos in *G*. *max* and *G*. *soja* will help to discover, examine and assess the pattern of VOZ protein sequence conservation in other plant species.

**Fig 1:** Vascular plant one-zinc-finger sequence logo of *G*. *max* and *G*. *soja*. Amino acid pattern depicts that they are highly conserved.

### Sub-cellular localization

Sub-cellular localization for GmVOZ and GsVOZ was initially predicted by using CELLOv.2.5 (http://cello.life.nctu.edu.tw/) and were found to be localized in nucleus. For confirmation, GmVOZ1-GFP and GsVOZ-GFP fusion proteins were expressed in tobacco leaves. GmVOZ1 and GsVOZ1 was specifically localized in the nucleus (Fig 2).

The article "Characterization of Vascular plant One-Zinc finger (VOZ) in soybean (Glycine max and Glycine soja) and their expression analyses under drought condition" was retracted in 2023. Reasons: a conflict of interest; concerns about the peer review; concerns about the authorship.

**Fig 2:** Sub-cellular localization of GmVOZ1 and GsVOZ1. Brightfield, fluoresence (GFP) and merged images of tobacco leaves infiltrated with *Agrobacterium*.

### Evolutionary and phylogenetic relationship of *VOZ* protein

Phylostratum analysis of *VOZ* genes identified the primitive ancestry as *VOZ* genes were present in *P*. *patens* (Bryophyte)- one of the early plant pedigree (Fig 3A). *VOZ* genes were existing in *A*. *comosus* (angiosperm), *A*. *thaliana*, *M*. *truncatula G*. *raimondaii*, *B*. *rapa*, *S*. *melongena*, *G*. *max*, *G*. *soja* and *P*. *trichocarpa* (dicotyledons), *Zea mays* and *B*. *distachyon* (monocotyledons). These results suggested that *VOZ* genes originated from early land plants’ phlyostratum and probable orthologous genes of *VOZ* are existing throughout plant kingdom. We also constructed ML tree to explore the deeper relationship of *VOZ* genes of 12 species. The prefixes, At, Gm, Gs, Pp, Pt, Gr, Sm, Zm, Br, Bd, Mt and Ac were used before the names of *VOZ* genes from *A*. *thaliana*, *G*. *max*, *G*. *sjoa*, *P*. *patens*, *P*. *trichocarpa*, *G*. *raimondaii*, *S*. *melongena*, *Z*. *mays*, *D*. *distachyon*, *M*. *truncatula* and *A*. *comosus*, correspondingly. The ML tree displayed that all 47 *VOZ* genes from 12 different species were classified into 7 clades. The clades were differentiated with different color schemes (Fig 3B). In this study, clade-1 (light-green color) and clade-3 (red-color) contained 13 genes each, followed by clade-7 (brown-color) having seven *VOZ* genes, clade-6 (orange-color) contained 2 while clade-4 (dark-green color) and clade-5 (purple-color) contained one each gene of *VOZ*. Clade-1/2 one contains genes from angiosperms and dicotyledons, clade-3 contains genes from dicotyledons, clade-5/6 contains genes from bryophytes and clade-4/7 contains genes form monocotyledons. We also found that *VOZ* genes of monocots and dicots were closely grouped to each other. Gene enlargement in *G*. *max* and *G*. *soja* can be detected in our phylogenetic analysis, as their eight pairs out of 12 were closely grouped to each other (Fig 3B). The paralogous pairs showed that *VOZ* genes underwent duplication event in their evolution resulting in gene family expansion.

**Fig 3:** Phylogenetic analyses of vascular plant one-zinc-finger (VOZ) from 12 different species. (A) The phylostartum analyses of *VOZ* gene family. (B) Phlyogenetic tree divided all 47 genes into seven clades. Bootstrap values were also mentioned near the node of each branch.

### Exon/intron and *cis*-element analysis

Exon/intron pattern in a single gene is related to its biological role. Gene structure analysis along with phylogenetic tree displayed that all *GmVOZs* and *GsVOZs* have three introns and four exons (Fig 4) and similar genes grouped close to one another in the same groups. We observed that all *GmVOZs* and *GsVOZs* exhibited conserved patterns of exon/intron structure even through gene duplication occurred a long time ago during evolution. Expression of genes is governed by promoter and by the binding of TF to *cis*-element present in the upstream region. PlantCARE database was used, to determine the *cis*-acting element in the upstream region of *GmVOZs* and *GsVOZs* gene. The result showed that *GmVOZs* and *GsVOZs* gene carried stress related *cis*-acting element in their promoter such as LTR (for low temperature), MYB, MBS (for stress and defense), ABRE and CGTCA-motif (for different stress response) and W-Box (fungal elicitor) repeats (Fig 5) [4–6].

The article "Characterization of Vascular plant One-Zinc finger (VOZ) in soybean (Glycine max and Glycine soja) and their expression analyses under drought condition" was retracted in 2023. Reasons: a conflict of interest; concerns about the peer review; concerns about the authorship.

**Fig 4:** Gene structure display of *G*. *max* and *G*. *soja*. Red-box represents untranslated and blue-box represents exon regions.

**Fig 5:** Putative *cis*-acting elements in a 2.0 kb 5’ flanking region upstream from the start codon of *GmVOZs* and *GsVOZs*.

### Expression profiling of *GmVOZs* and *GsVOZs*

Gene expression profiling foretells the biological role of a gene; hence we investigated the expression of *GmVOZs* and *GsVOZs* in Williams-82 and W05, respectively. All genes were used to assess the tissue specific transcript abundance levels by qRT-PCR in roots and leaves at seedling stage, green pods, flower, seed 10, 21, and 35 days after flowering. These results indicated that *VOZ* might play functional roles in different developmental stages of soybean. Moreover, all studied genes had relatively higher transcript level in roots revealing their role with limited functional divergence during evolution (Fig 6). Analyses of *GmVOZs* and *GsVOZs* gene expression under PEG6000 was also performed in this study. The responses of all studied genes were observed at different time points i.e., 0h, 1h, 3h, 6h after treatment via qRT-PCR. All studied genes had higher transcript level as compared to control (0h) at various time intervals for PEG6000 treatment (Fig 7). Together with these observations, *GmVOZs* and *GsVOZs* showed obvious resistance against PEG6000 treatment advocating that these genes are possible candidates for breeding drought resistant soybean cultivars.

**Fig 6:** Expression analysis of *GmVOZs* and *GsVOZs* genes at different developmental stages in specific organs. Leaves (L), Roots (RT), Green Pods (GP), Flower (FL), Seed 10, 21, 35 days after flowering.

**Fig 7:** Expression pattern analyses of *GmVOZs* and *GsVOZs* under PEG6000 treatment estimated by qRT-PCR analyses. The error bars show standard deviations.

The article "Characterization of Vascular plant One-Zinc finger (VOZ) in soybean (Glycine max and Glycine soja) and their expression analyses under drought condition" was retracted in 2023. Reasons: a conflict of interest; concerns about the peer review; concerns about the authorship.

### Chromosomal distribution, gene duplication and synteny analysis

The studied *GmVOZs* and *GsVOZs* were mapped to their corresponding chromosomal loci. The results exhibited that the chromosomes contained only single *GmVOZ* and/or *GsVOZ* gene. The uneven distribution denotes that the gene loss might have taken place during evolution.

To explore the locus relationships among *GmVOZs* and *GsVOZs* genes, we identified the orthologous/paralogous gene pairs for the cultivated and wild soybean. Synteny analysis showed that several gene loci are highly conserved (Fig 8). A total of 14 orthologous/paralogous gene pairs were identified, of which all studied genes were attributed to segmental or whole genome duplication (WGD) to form paralogous gene pair between both species. During the process of evolution, gene pairs can undergo functional divergence which can result in non-functionalization (when two duplicated genes acquires a mutation in regulatory or coding regions that renders the gene non-functional), sub-functionalization (directs specific function of gene expression), or neo-functionalization (when one of the two duplicated genes acquires a mutation in regulatory or coding regions resulting in novel and useful function of gene). *Ka/Ks* values were calculated to determine the extent and nature of selection pressure on these duplicated gene pairs. It has been established that *Ka/Ks* = 1 indicates pseudogenes because of neutral selection, *Ka/Ks* > 1 represents positive selection of accelerated evolution, while the ratio of *Ka/Ks* < 1 exhibits the ability for genes duplication for purifying selection. In this study, we found that all *GmVOZs* and *GsVOZs* genes showed *Ka/Ks* values less than 1 (S3 Table), anticipating that soybean *VOZ* genes were subjected to purifying selection pressure with limited functional deviation because of WGD and segmental duplication. The *Ka* and *Ks* divergence values exhibited that for 14 duplicated gene pairs.

**Fig 8:** Gene duplication among *GmVOZs* and *GsVOZs* gene. Blue line indicates orthologous/paralogous pairs. Gm01 to Gm20 indicates the chromosomes of *G*. *max* and Gs01 to Gs20 represent the chromosome of *G*. *soja*.

## Discussion

Present yield grain trends in important crops are insufficient to meet the requirements of global population of ~ 9 billion by 2050. This is further challenged by climate change which is anticipated to get worse with extreme weather events and it has been well established that, water stress limits growth, development, and productivity in crop plants [1]. The present genomics landscape of crop plants has been revolutionized, courtesy next generation sequencing technologies which offer sequencing information up to many manifolds. The availability of genome assemblies for soybean [1] creates new opportunities for more precise genome-wide studies in soybean. Several experiments have been performed to explore the role and biological function of *VOZ* genes in different crop plants [8, 10–12, 15, 16]. However, no systematic analyses of *VOZ* genes in *G*. *soja* in comparison with *G*. *max*, has been reported till date. In present study, we conducted analyses of *VOZ* genes in cultivated (*G*. *max*) and wild (*G*. *soja*) species of soybean. Ours is the first study to investigate the evolutionary relationships, gene duplication and selection pressure on *GmVOZs* and *GsVOZs*. Recent advancement in soybean genome sequencing made it possible to conduct present exploration [1, 17]. This study will be helpful in laying a foundation for further work.

The article "Characterization of Vascular plant One-Zinc finger (VOZ) in soybean (Glycine max and Glycine soja) and their expression analyses under drought condition" was retracted in 2023. Reasons: a conflict of interest; concerns about the peer review; concerns about the authorship.

### *GmVOZs* and *GsVOZs* genes show evolutionary conservation

We classified *VOZ* genes from bryophytes, angiosperms, dicots and monocots. Phylostratum analysis of *VOZ* gene family revealed that the primitive plant pedigree as *VOZ* genes were present in *P*. *paten* (bryophytes), suggested that *VOZ* genes originated from non-vascular plants phylostratum and potential orthologous genes are present throughout kingdom plantae [26]. The existence of *VOZ* genes in each selected species, with nine *VOZ* genes from *B*. *rapa*, six *VOZ* genes from *G*. *max* and *G*. *soja*, and only two genes from *P*. *patens*, revealed the evolutionary conserveness of *VOZ* genes and these genes experienced expansion in higher plants. Furthermore, *GmVOZ* and *GsVOZ* genes represented close relationship, strengthening the fact that both species shared common ancestor [2]. Sequence logos, for AARs were highly conserved in *G*. *max* and *G*. *soja* at N and C termini showing that *VOZ* genes are evolutionary conserved which might be helpful to know the outline of VOZ protein sequence conservation in other species.

Promoter sequences of *GmVOZ* and *GsVOZ* genes had nearly same distribution of *cis-*elements related to stress responses. The *cis-*elements such as LTR, MYB, MBS, ABRE, CGTCA-motif and W-Box were identified in both studied species of soybean. The presence of these *cis*-elements with specific features depicted the predicted functions in plant growth, development, biotic and abiotic stress resistance. Exon-intron structure is important that may be contributed by insertion/deletion events. Several studies reported extensive gain or loss of introns during eukaryotic diversification. Gene structure analysis exhibited that duplicated genes have similar exon-intron pattern, whereas, intron length differs among different genes showing that intron length may play crucial roles in the functional diversification of *GmVOZ* and *GsVOZ* genes. Introns also play important role for the evolution of different plant species [27]. Here, we found that all *GmVOZ* and *GsVOZ* genes had three introns showing that both *G*. *max* and *G*. *soja* were newly evolved with fewer introns, which supported previous studies that intron numbers decreased with the passage of time [28] and suggested that newly evolved species have fewer introns as compared with primitive ones [27]. Gene structure of *GmVOZs* and *GsVOZs* were extremely similar, showing that these genes were highly conserved. Moreover, introns experienced weak selection pressure and presence of a greater number of introns were thought to have gained novel functions during evolution.

The article "Characterization of Vascular plant One-Zinc finger (VOZ) in soybean (Glycine max and Glycine soja) and their expression analyses under drought condition" was retracted in 2023. Reasons: a conflict of interest; concerns about the peer review; concerns about the authorship.

### *GmVOZs* and *GsVOZs* gene expression are regulated by drought stress

The results of ours study demonstrated that *GmVOZs* and *GsVOZs* have higher transcript abundance in leaves and roots at seedling stage, showing the positive role, that these genes may play in plant growth and root development. *VOZ* genes are likely to respond in an ever-changing environment and are involved in plant growth and development [8, 17, 29]. *AtVOZ1* and *AtVOZ2* redundantly support flowering in photoperiod pathway [10]. In rice, *OsVOZ1* and *OsVOZ2* were shown to be rapidly induced in response to water stress [31] Similar results were obtained by Li et al. and Dey et al. [17, 30]. However no systematic study of *VOZ* genes in *G*. *soja* has been reported till to date. The expression of *GmVOZ* and *GsVOZ* genes can considerably be upregulated by abiotic stress such as PEG. Together with these outcomes, we conclude that *GmVOZ* and *GsVOZ* genes might be instrumental for breeding drought tolerant soybean.

### Gene duplication and selection pressure

Tandem duplication events happen when two or more genes are positioned on same chromosome, whereas, segmental or WGD events occurr between the chromosomes. Tandem duplications support increment in introns and can generate novel genes [31] however, we did not find evidence of tandem repeat in this work. All gene pairs were associated with segmental or WGD. Many gene families expanded more in plants as compared to other eukaryotes, indicating that these expansions were associated with environmental and selection pressures. The sequence based tools assist to study the organization, evolution and syntenic relationships of genomes. By using linkage maps, synteny of various species can be compared and in general, closely related species shows higher synteny level and this syntenic level decreases with growing phylogenetic distance [32]. Fourteen paralogous/orthologous gene pairs within and between *G*. *max* and *G*. *soja* were identified. The *Ka/Ks* values showed that soybean *VOZ* genes underwent strong selection pressure with limited functional deviation arising from whole genome and segmental duplication. To estimate the environmental and selection pressure, *Ka* and *Ks* substitution rates were calculated. In general, *Ka/Ks* < 1, *Ka/Ks* > 1 and *Ka/Ks* = 1 indicate purifying selection, positive selection and neutral evolution, correspondingly [4, 6]. In current work, we observed that *Ka/Ks* values of *GmVOZ* and *GsVOZ* genes were < 1 suggesting that *GmVOZ* and *GsVOZ* genes experienced strong purifying selection pressure.

The article "Characterization of Vascular plant One-Zinc finger (VOZ) in soybean (Glycine max and Glycine soja) and their expression analyses under drought condition" was retracted in 2023. Reasons: a conflict of interest; concerns about the peer review; concerns about the authorship.

## Conclusion

In this study, six genes each of *GmVOZs* and *GsVOZs* were investigated and were further split into four major groups on the basis of phylogenetic analyses. Sequence logos analyses between *G*. *max* and *G*. *soja* amino acid residues showed higher conservation. Presence of abiotic stress *cis*-elements in the promoter regions of *GmVOZs* and *GsVOZs* clearly showed their role in tolerance against environmental stresses. Collinearity analysis revealed that the studied genes underwent purifying selection pressure. Gene expression experiment results showed the studied genes differentially expressed under normal and drought stress conditions. The present work was the first systematic analysis and comparison between *G*. *max* and *G*. *soja*. These outcomes provide a foundation for further exploring the functions of *GmVOZs* and *GsVOZs* in plant abiotic stress responses.

## Supporting information

S1 Table Oligonucleotide sequences and enzymes used in present study. (DOCX)

S2 Table Biophysical properties of *GmVOZ* and *GsVOZ*. (DOCX)

S3 Table Gene orthologous/paralogous and *Ka/Ks* value estimation. (DOCX)
